The article "Research on Impulse Power Load Forecasting Based on Improved Recurrent Neural Networks" was published in 2022. Journal: Comput Intell Neurosci.

# Research on Impulse Power Load Forecasting Based on Improved Recurrent Neural Networks

**DOI:** 10.1155/2022/2784563

**Published:** 2022-04-23

**Authors:** Chenyang Feng, Kang Xu, Haoyun Ma

**Affiliations:** College of Electrical Engineering & New Energy, China Three Gorges University, Yichang, Hubei 443002, China

## Abstract

Deep learning is good at extracting the required feature quantity from the massive input information through multiple hidden layers and completing the learning through training to achieve the task of load forecasting. The impulse power load data contain a lot of noise, burrs, and strong randomness. As an improved recurrent neural networks, the output of long short-term memory (LSTM) network is not only related to the current input, but also closely related to the historical information, which can effectively predict the impact power load. An impulse power load forecasting model based on improved recurrent neural networks is proposed. To solve the training difficulties caused by deep networks, database is divided into training data set and test data set. To accelerate running speed and improve accuracy and reliability, parameter setting in deep learning neural network is analyzed. The proposed load forecasting model is verified by simulation and compared with the existing methods. Taking the average relative error as the standard, the effectiveness of the proposed model for the forecasting of impulse power load connected to the bus is verified.

## 1. Introduction

Grid load forecasting refers to periodic load forecasting for power equipment such as generator sets, power users, and power loads, so as to make reasonable planning to ensure the safe and stable operation of power system. Short-term load forecasting (STLF) is one of the important tasks of energy utilization, power planning, dispatching, and other management services [1–4]. In fact, considering the different operation laws and performance of each power system, on the premise that the transmission accuracy requirements are not discounted, and considering the different influencing factors (including natural environment, human development, social change, etc.), if we can accurately predict the change and fluctuation of power load in the future, it will promote planned energy and power use management.

STLF is beneficial to the preadjustment of power grid operation mode and the arrangement of unit maintenance plan [3, 4]. It can save coal and fuel and is conducive to the compression of power generation cost, which is conducive to the rational development of energy and the formulation of construction plan.

At present, the research direction of power load forecasting mainly focuses on the utilization of algorithm, the establishment and application of mathematical model, and the determination of main influencing factors [2, 4]. Due to the strong nonlinearity and many random factors of power short-term load, the previously proposed load forecasting theory has shown limitations and deficiencies. The development of new technologies, new ideas, and new methods is the driving force for the long-term and sustainable development of power load forecasting.

With the implementation of energy conservation and emission reduction policies, new energy power plants and ultrahigh voltage (UHV) power grid system are developing rapidly, with a wide variety of power sources, so the load change is more difficult to predict. At the same time, alternating current (AC) and direct current (DC) in UHV are very complex, and the operation and maintenance of power grid is more difficult and faces great challenges. In new energy power stations, wind power plants and photovoltaic power generation have sprung up under the incentive of policies. However, due to the uncertainty of wind power and solar power generation, the power grid will be violently turbulent. Therefore, how to realize the impact load forecasting of multiple power sources is an urgent problem to be solved.

## 2. Characteristic Analysis of Impulse Power Load Forecasting

In some areas, due to the existence of large iron and steel enterprises, the impact load accounts for the majority of the overall load, which seriously reduces the accuracy of local load forecasting results. On the premise that some breakthroughs have been made in each new load model, at present, the development of power market is gradually restricted by the accuracy of power system load forecasting and the forecasting state gradually tends to saturation [5]. The application of artificial intelligence in STLF can effectively improve the forecasting accuracy under complex environmental factors. Adding deep learning to power system, STLF can form a higher level of deep intelligence, which can not only manage the security of transmission system, but also play a key role in cost budgeting and power distribution.

Internal and external characteristics are collectively referred to as power load characteristics. The law that the load power changes with the frequency of the load system or the voltage on the load terminal is called the internal power load characteristic, which can be divided into frequency characteristic and voltage characteristic. The inherent load characteristics are mostly used for the analysis of system stability. Usually, the load curve is often used to describe the power load changing with time and reflect the change law of load data in a period of time [6]. However, the daily load curve of power grid in iron and steel impact area is often irregular and even cannot find any regularity all day.

There are various types of steel load, usually including stainless steel, milk line, electric arc furnace, oxygen production, section steel, etc.; and it has heavy single line load, ranging from 30 MW to 80 MW. In the power system load in a region, the impact load capacity of iron and steel enterprises is huge, with high randomness and poor regularity. Some enterprises need to arrange the production plan according to the preferential section of peak and valley prices. Sometimes the production plan will be adjusted due to events, and the accuracy of load forecasting will be greatly reduced.

## 3. LSTM Model

Long short-term memory (LSTM) [7–9] is a variant form developed and improved by recurrent neural networks (RNN). The structure of “gate” of LSTM neural network is used to control the state of nucleus. A selective gate function information through which cell core states can be added or removed. The ancestor macros form a set of cyclic subarrays called memory blocks. The memory or forgetting of key node information is selected to realize the combination of long-term memory and short-term memory. This improves the spatiotemporal task which is difficult to be controlled by RNN artificially. The “gate” of LSTM neural network is utilized by a sigmoid neural network layer through point-to-point multiplication operation.

An output value of “0” for the sigmoid layer means no information can be passed, but a value of “1” means all information can be passed. LSTM neural network has three gate structures, including “input gate,” “output gate,” and “forgetting gate.” They are used to control and protect the state of the core of the unit.  Figure 1 shows the LSTM structure.

The detailed derivation of the arithmetical expression of LSTM neurons follows. Let us set the time variable to *t*. The input variable of LSTM (long short-term memory recurrent neural network) set as the sequence input of time *t* is *x*_*t*_, the LSTM output of time *t* − 1 is *h*_*t* − 1_, and the gating state quantity of time *t* − 1 is *s*_*t* − 1_. LSTM output *t* is the output value *h* of LSTM at time *t*. State *s*_1_ of the door control unit at time *t*. In LSTM, the oblivion gate works by turning the last moment's HT. The *x*_*t*_ at this time is regarded as the input to the sigmoid layer. It outputs values between 0 and 1 and sends them to *s*_*t* − 1_. Determining the influence of *x*_*t*_ on its *s*_*t*_ is within the function range of the input gate. It is the function of the output gate to control the influence of *s*_*t*_ on *h*_*t*_. The arithmetic expressions of forgetting gate, input gate, and output gate are as follows:

(1) $$\begin{array}{c} i_{t}=\sigma \left(W_{i}\left[h_{t-1},x_{t}\right]+b_{i}\right),\\ f_{t}=\sigma \left(W_{f}\left[h_{t-1},x_{t}\right]+b_{f}\right),\\ O_{t}=\sigma \left(W_{o}\left[h_{t-1},x_{t}\right]+b_{o}\right), \end{array}$$

where *f*_*t*_, *i*_*t*_, and *o*_*t*_ represent the calculation results of LSTM forgetting gate, LSTM input gate, and LSTM output gate state, respectively.

*W*_*f*_, *W*_*i*_, and *W*_*o*_ are the weight matrices of LSTM forgetting gate, LSTM input gate, and LSTM output gate, respectively. *b*_*y*_, *b*_*i*_, and *b*_*o*_ are bias items of LSTM forgetting gate, LSTM input gate, and LSTM output gate, respectively. The final output of the LSTM is determined by the output of the output gate and the output of the cell state.

(2) $$\begin{array}{c} {\hat{s}}_{t}=\tan\;h\left(W_{s}\cdot \left[h_{t-1},x_{t}\right]+b_{s}\right),\\ s_{t}=f_{t}\cdot s_{t-1}+i_{t}\cdot {\hat{s}}_{t},\\ y_{t}=o_{t}\cdot \;\tan\left(s_{t}\right), \end{array}$$

where *s* represents the input unit state of time *t*, *W*_*s*_ is the weight matrix of the input cell state, *b*_*s*_ is the offset term of the input unit, and tan *h* is the activation function type.

## 4. Deep Learning Adaptability of Bus Load Forecasting Problem

In the early years, foreign experts and scholars have done the work of substation bus load prediction [10–12]. Due to the increasing demand of power grid dispatching and the mature development of dispatching technology, bus load forecasting is also widely used to solve the security and stability analysis of power system, reactive power optimization of power plant, and system dynamic state estimation.

Accurate bus load prediction is a prerequisite for the safety and stability of power system. In order to adjust generation plan reasonably, realize safety check, and implement energy-saving generation, it is very important to improve the accuracy of bus load forecast.

### 4.1. Characteristics of Bus Load Prediction

Compared with the traditional system load forecasting, bus load forecasting has its own features:

1. As the basic unit of system load prediction, bus load prediction has frequent changes compared with system load prediction. It has the characteristic of small prediction base, and the cardinality is much lower than the system load, which leads to the error of bus load prediction and difficult to improve the prediction accuracy.
2. Bus load prediction nodes are large, and the number of regional buses is large. For Laiwu power grid, there are 11 220 KV substation busbar loads to be processed. Each substation has a dual bus connection, resulting in 22 predictive nodes.

Large proportion of power grid in Laiwu area is connected to steel load. Its impact is very strong and difficult to find rules, and uncertain production plans and maintenance plans make local load forecasting work more difficult.

### 4.2. Bus Load Forecasting Process

The busbar load forecast of the substation shall be reported again after adjustment by the provincial company and the prefectural company. Weather, politics, social activities, holidays, and other factors affecting bus load change should be considered when adjusting. According to the accumulated historical load changes, the correlation between various indicators and load changes is comprehensively analyzed, and the factors affecting load changes and historical load data are used as the input of the model. The target load, that is, the load value to be predicted, is the output target of training.

As mentioned above, deep learning is good at extracting required feature quantities from massive input information through multiple hidden layers. Finally, the training completes the task of load prediction, especially for short-term power load prediction. Load data are values that change with time. It is both nonlinear and sequential. In the process of load forecasting, the problem of long-term dependence on historical information often appears. The application of LSTM neural network in load prediction can prove its effectiveness theoretically. As a variant of RNN, the output of LSTM is not only related to the current input but also closely related to historical information. Therefore, LSTM has strong applicability in time series. In addition, the impact load data of steel studied in this article contain a lot of noise, burrs, and strong randomness. In theory, mathematical statistics are not as good as machine learning.

To sum up, deep learning method is suitable for charge prediction. Deep learning deals with the time series of power load itself and the nonlinear relationship between various influencing factors and charge.

## 5. Case Study

### 5.1. Experimental Data Sample

According to the preliminary investigation, the large steel enterprise is supplied by a number of substations with different capacities. In order to carry out this analysis, a total of 35,040 load data of several typical Laiwu 220 KV busbars connected to the largest energy consuming equipment or production line in 2018 were selected as the data set for simulation. A 15-minute interval is taken as a sampling interval, and 96 intervals of load data are taken for 24 hours per day. The change of load data needs to consider its busbar load operation mode and maintenance plan adjustment, seasonal change characteristics. Usually, 1–3 months is used as the interval time of model training. Due to the particularity of the historical load of the busbar in the area connected to large steel enterprises, the training time of the model is selected from 2 to 3 months. According to the typical seasons, the sample data set is the historical load data from April to May, June to July, and October to December.

### 5.2. Evaluation Indicators of Forecasting Method

Different power load forecasting models and methods usually have different performance. In order to compare the advantages and disadvantages of various prediction methods and the performance of models, it is important to design reasonable and feasible evaluation indexes for quantitative prediction performance. In this article, mean absolute percent error (MAPE) and root mean square error (RMSE) are selected as two reference indexes to judge accuracy.

The average absolute error evaluates the average absolute error between the predicted value and the real value, and its value range is [0, +*∞*). The smaller the value is, the better the model fitting effect is. The model is perfect if the error is zero.

(3) $$\begin{array}{c} \text{MAE}=\frac{1}{n}\overset{n}{\underset{i=1}{\sum }}\left|f_{t}\left(i\right)-f_{p}\left(i\right)\right|, \end{array}$$

where *f*_*t*_(*i*) represents the simulated predicted value at time *I*, *f*_*p*_(*i*) represents the real load value at time I, and *n* indicates the input of load data.

Mean absolute percentage error. The reason why the mean absolute percentage error can describe the accuracy is that the mean absolute percentage error itself is often used to measure the accuracy of the statistical indicators, such as the prediction of time series.

The size of the mean square error is calculated from the sum of the squares of the errors. It measures the error between the predicted value of a model and the actual value of the load by means of the mean square error. The value is between [0, +*∞*), and the smaller the index value is, the better the model effect is.

(4) $$\begin{array}{c} \text{MAE}=\frac{1}{n}\overset{n}{\underset{i=1}{\sum }}{\left(f_{t}\left(i\right)-f_{p}\left(i\right)\right)}^{2}. \end{array}$$

The root mean square error (RMSE) of large error has a stronger influence on the index, and the index will be more sensitive. This is a good indicator of the accuracy of the measurement. Therefore, RMSE is widely used as a standard for error prediction. The value range is [0, +*∞*). The smaller the value of the exponent, the better the effect of the model.

(5) $$\begin{array}{c} \text{RMAE}=\sqrt{\frac{1}{n}\overset{n}{\underset{i=1}{\sum }}{\left(f_{t}\left(i\right)-f_{p}\left(i\right)\right)}^{2}}. \end{array}$$

In the essence of mathematical expression, mean absolute error, relative error, absolute error, and MAPE are the same. They are linear expressions of the predicted deviation from the true value. In this article, RMSE is selected as the performance evaluation index of the prediction method.

The error evaluation standard in this article is based on the load prediction evaluation standard of Shandong Electric Power Company of State Grid.

The formula for calculating the accuracy of the average daily load forecast is as follows:

1. Reference error of single bus load in period K
2. Reference error = (actual load − predicted load)/load reference value*∗*100%
3. The load reference value is 305 MW temporarily
4. Regional errors of all busbars in *k* period
5. Area error = root mean square of reference error of all buses
6. Accuracy of all busbars at all times of a day
7. Accuracy = (1 − root mean square of regional error for all time periods)*∗*100%

### 5.3. Deep Learning Model

The programming and simulation work in this article is based on MATLAB R2018b platform. The so-called network and deep learning algorithm is a deep learning toolkit from MATLAB. The historical load data used in load forecasting have both long-term dependence and short-term dependence of time series, and the influence of other aspects cannot be ignored. This chapter uses historical load database and influence factor processing to carry out the learning and prediction work based on deep learning network.

#### 5.3.1. Model Building

Because LSTM has a memory structure, it can well reflect the load data relationship in time series. When using deep learning LSTM networks in extremely short-term load prediction scenarios, an important step is to preprocess a large amount of historical load information. This solves the training difficulties caused by deep networks and many parameters. This chapter divides database into training data set and test data set, with a ratio 7 : 3. The former is used for deep learning network model learning process, and the latter is used for model performance test after training.  Figure 2 shows the flowchart of load forecasting network based on LSTM.

#### 5.3.2. Input and Output

In order to better meet the load forecasting demand of large steel enterprises, on the basis of general power load forecasting, the high sensitivity of industrial load to electricity price is taken into account. Large steel mills use lower loads during the day, when the electricity price is high, than at night at the cutoff point of the electricity price change at 8 a.m. The load it uses is significantly reduced. At the same time, steel load and steel market price changes are positively correlated. When the steel market booms, the steel load will increase accordingly. On the contrary, when the steel market downturn, steel load will be reduced accordingly. After a thorough examination, historical load data, changes in steel futures levels, date types, electricity price fluctuations, and weather changes are taken as influencing factors for load forecasting. Based on the historical data input in the LSTM network model, the influencing factors of the predicted date were used as the feature input template. Because every day there are points with large load fluctuations, the timing and amplitude of these points are characterized by very irregular. The bus load forecasting in Laiwu city can be used for reference. Two sets of input feature sets for load forecasting are summarized after considering various realistic situations. The former feature set network inputs the load data of 96 points in the 7 days before the forecast day and the date type, temperature, electricity price, steel price, and other information of the forecast day. The output data are the forecast daily load data of 96 points. The input data of the latter feature set network are the load data of 96 points 1 day before the forecast day and the date type, temperature, electricity price, steel price, and other information of the forecast day. The output data are the 96-point load data of the day to be predicted. The input feature set is shown in Table 1.

Input 1 is the historical load factor. The historical load information input of model 1 is 96 points of load data per day for 7 days starting from the day before the forecast date. The input of historical load information in model 2 is the load data of 96 points on the day before prediction. Input 2 indicates the date type (holiday or not) of the day to be predicted. Input 3 is meteorological condition, which mainly represents the 96-point fluctuation data of temperature on the day to be predicted. Input 4 is only reflected in Model 2, which is the weather condition of the day to be predicted. Input quantity 5 is the fluctuation of electricity price, which inputs the electricity price in different time periods of each day according to the price of peak and valley. Inputs 6-7 are the price change of steel futures, which shows the price fluctuation of rebar and H-beam.

Since the deep LSTM network has a storage unit, the loading data structure information can be encoded in the parameters of the LSTM network to preserve the timing of data. Let the historical load and influence factor data set be the matrix *X* of *m* × *n*.

(6) $$\begin{array}{c} X=\left[\begin{array}{cccc} X_{11} & X_{12} & \cdots & X_{1n}\\ X_{21} & X_{22} & \cdots & X_{1n}\\ \vdots & \vdots & \ddots & \vdots \\ X_{m1} & X_{m2} & \cdots & X_{\text{mn}} \end{array}\right]. \end{array}$$

In the matrix, *M* is the step size of the training sample information, *n* is the number of input characteristic information, and *X*_*ij*_ represents the JTH characteristic information of the *i*^th^ input value. A day of data contains 96 lines. Take 1 day's data as the previous progress. The forward progress length of the longitudinal dimension input is 7, and the data volume of 7 days is entered into the model simultaneously. The 672*∗*12 matrix of the output data and the 96-point load data on the predicted day are the output of the LSTM network model.

#### 5.3.3. Network Structure of the Model

In order to create a deep learning network structure suitable for different topics, we need to conduct centralized testing and debug the network parameters to the best, so that the network effect can meet the needs. When the number of layers and hidden units of LSTM network is too small, that is, the number of neurons in the network is too small, the network model to model building and feature extraction will not occupy a great advantage. When the number of neurons are too large, the learning efficiency of the network will decrease and over-fitting phenomenon will occur. Online learning time will also increase significantly. Therefore, when considering the STLF work in reality, the parameters of LSTM network used should be reasonably selected. Many experiments are carried out in this article, and the best parameters are selected according to the results.  Figure 3 shows the LSTM network structure.

### 5.4. Simulation and Verification

#### 5.4.1. Simulation Settings

In the process of building LSTM neural network, the neural layer and input layer of the network and the expression of Loss need to be defined first. Optimizer minimizes loss. The appropriate training data should be selected first to train the model. Selecting appropriate network parameters during training can accelerate the running speed of recursive neural network in deep learning and improve the accuracy and reliability of load prediction. The analysis of parameter setting in deep learning neural network is as follows:

1. Input layer and output layer: the number of nodes in the input and output layers is related to the type of historical power load data and the type of influencing factors. In this article, the data set used in the simulation was selected for a 15-minute sampling interval and 96 load data per day. There are many factors that affect the prediction of power load. On the basis of the preprocessing of the historical load analysis, the data are normalized and the main factors affecting the load are taken as the input of the model.
2. Based on the analysis of the historical load prediction accuracy of bus lines in Laiwu area, the bus lines connected with steel shock load are divided into two types of research. The first bus has a certain steel impact load. Taking bus no. 2 of Shuanglong Station and bus No. 1 of Fangxia Station as examples, certain periodic regularity can be found, and the historical prediction accuracy is fair. The second bus is almost fully loaded with steel shock load. It is difficult to find cyclical regularity and is very sensitive to changes in the production plans of iron and steel enterprises. The accuracy of historical load prediction is not ideal for the #2 bus line of Gangcheng station and #2 bus line of Huihe Station.
3. On the basis of the above model input study, this article proposes two network models to improve the accuracy of load prediction of impact load bus of access steel.
4. First, the historical load factor of the first type model selects the load data of the day to be predicted, the date type of the day to be predicted, the 96-point temperature data of the day, the weather type of the day to be predicted, electricity price fluctuation data, and steel price data.
5. Second, in the second type of model, the historical load factor selects the load data of the 7 days before the forecast day, the date type of the forecast day, the 96-point temperature data of the same day, electricity price fluctuation data, and steel price data.
6. According to a lot of simulation experience, the first type of model performs better in bus load prediction which is more sensitive to external factors. The typical characteristics of this kind of busbar are that it is more affected by the change of production plan of iron and steel enterprises, it is difficult to find the periodic law, and the accuracy of historical load prediction is low. The second model performs better in bus load prediction with stable steel generation and production process. This kind of bus has a certain impact load of steel, and its historical regularity of load data is easier to grasp than the former one.
7. The number of nodes in the hidden layer is based on other researchers' research experiments. More hidden layers have better network training effect, but the training time will be longer. Since the training example in this article is a short-term charge prediction example, multiple hidden layers can be selected to deal with more complex cases. The actual network structure usually has no fewer than 100 neural units.
8. Learning rate of deep learning network is the convergence time of control function. It depends on the network read value and weight. With the increase in learning rate, the model training speed is accelerated. The stronger the effect of corresponding output error on parameters is, the more likely it is to oscillate and diverge. The learning rate decreases, the model training speed slows down, and the function is prone to over-fitting and over-converging.
9. Time step determines the learning span, that is, the input data depend on several consecutive input data.
10. The training of loss function (Loss) is to reduce the Loss value of training set and verification set. When the loss value is lower than a certain threshold or reaches over fitting, the training ends.
11. Training duration (EPOCHS): by reducing or increasing the number of trainings, under-fitting or over-fitting can be avoided.

Generalization ability of deep learning model is also a problem that needs to be considered in model training. Generalization ability refers to the ability of deep learning model to respond reasonably to updated data. A good model must have strong generalization ability. It is common to find that the model is too fit or not trained enough in the process of model training. Model over-fitting reflects the generalization ability of the model. In the case of too many training times or too little training data, the deep learning model can fit the training set data well. It cannot fit the test set data efficiently and well. In order to solve this problem, it is necessary to plan the duration and cycle of model training reasonably and effectively. Training must be stopped before the inflection point of test loss and training loss occurs.

According to the simulation experience, relatively small learning rate is better to ensure the stability of the system. The selection range of learning rate is between [0.01, 0.8]. This is to observe the variation trend of training set and validation set error and the accuracy of load prediction results. Through a large number of simulation experiments in the early stage, the parameters of the deep learning model were constantly adjusted and finally the learning rate was set as 0.01 and the training duration as 800. In this LSTM network structure, the hidden layer is set as three layers, namely three LSTM layers, each layer is set with 150 hidden nodes, namely 150 long short-term memory units. The last layer is the full connection layer, which serves as the output layer of the model.

#### 5.4.2. Simulation Results

Two models are used to predict the typical bus, respectively, and the results are as shown in Table 2.

Taking Gangcheng station #2 bus line as an example, the variation of the load prediction model on the forecasting error in 7 days is analyzed, which is shown in Table 3.

Considering the changes of bus load in the area of steel shock load, such as operation mode adjustment, maintenance plan, equipment start-up and maintenance of iron and steel enterprises, and seasonal influence, three data sets are set according to the typicality, which are the historical load data sets of each bus in Laiwu area from April to May, from June to July, and from October to December in 2018, respectively. It carries on training and testing work with this input model. The results are compared with the current load forecasting method of Laiwu power grid obtained from preliminary investigation, as shown in Tables 4–6.

The existing regional forecasting method only considers the correlation between time factor and load. After the forecast, operators need to further adjust the forecast results according to the production plan of steel enterprises to obtain the load prediction curve. The internal and external factors affecting load variation including the characteristics of large steel enterprises are not considered. Therefore, the load prediction accuracy of the deep learning LSTM prediction algorithm used in this article, which considers a variety of influencing factors, is significantly improved compared with the traditional method.

The load prediction accuracy of Shuanglong bus No. 2 and Fangxia bus No. 1 increased by about 1%. The load carried by the busbars of the two substations fluctuates less than 50 MW. It has some regularity. Compared with the other three data sets, the improvement in the accuracy of Huihe 2# bus shows obvious difference, which is related to the fluctuation of quarterly load. When the fluctuation is small, the accuracy will be significantly improved, and when the fluctuation is large, the accuracy will be slightly improved. With regard to Gangcheng Station no. 2, the busbar carries the load of Dongling station and Section steel station of large iron and steel enterprises, so the load fluctuates greatly. In some special conditions, the instantaneous load fluctuation can exceed 100 MW, so the prediction method alone cannot meet the requirement of improving the prediction accuracy.

To further improve the accuracy of the prediction, the following direction of production planning and manual intervention is considered:

1. For the rapid load changes caused by the impact load superposition of large steel enterprises, special workers need to refer to the production process and production plan of steel mills. It modifies or replaces wave point data with boundary values.
2. Sudden load changes caused by accident trip and maintenance of electrical equipment require field operators to revise the prediction results according to the actual situation.

## 6. Conclusions

At present, the forecasting of steel impact load is mainly STLF, and the identification of influencing factors is mainly limited to production plan, maintenance plan, and other factors related to the production of iron and steel enterprises. Due to the complexity and high nonlinearity of influencing factors in the process of STLF, the traditional forecasting method has simple mathematical model, difficult to adjust parameters flexibly, and poor adaptability and relatively weak ability to reflect load changes. Therefore, it is difficult to further improve the prediction accuracy.

Compared with the mainstream artificial neural network algorithm and support vector machine algorithm, the impulse power load forecasting based on improved recurrent neural networks (LSTM forecasting algorithm based on deep learning network) proposed in this article can improve the accuracy of load forecasting. This point also directly proves the advanced nature of deep learning and its characteristics for dealing with load forecasting problems.

Nonlinear load is one of the main pollutants affecting the quality of power system. The characteristic power of high fluctuation load changes rapidly, and the load curve presents sawtooth wave. When the amplitude of load change is larger than the system capacity, it will cause continuous oscillation of system frequency and large fluctuation of voltage, which will have an adverse impact on the power system. The regularity of this kind of system load is usually very poor. It is very important to improve the accuracy of this kind of load forecasting. Future research will focus on this aspect.

## Figures and Tables

**Figure 1:** LSTM neuron structure.

**Figure 2:** Load forecasting network based on LSTM.

**Figure 3:** LSTM network structure diagram.

**Table 1:** Input feature set.

Input sequence no.	The input character description	
	Model 1	Model 2
1	96-point daily load curve for 7 days before forecast	96-point daily load curve from 1 day before the forecast date
2	Date type of the day to be predicted	Date type of the day to be predicted
3	96-point temperature fluctuation on the predicted day	96-point temperature fluctuation on the predicted day
4	—	Weather conditions for the forecast day
5	96-point electricity price on forecast date	96-point electricity price on forecast date
6-7	Forecast the day before the price trend of steel	Forecast the day before the price trend of steel

**Table 2:** Typical bus load forecasting accuracy.

Forecasting object	Model 1 (%)	Model 2 (%)
Shuanglong station #2	97.07	95.98
Fangxia station #1	93.98	92.30
Gangcheng station #2	93.59	92.47
Huihe station #2	94.59	93.54

**Table 3:** Gangcheng station #2 load forecasting accuracy.

	Model 1 (%)	Model 2 (%)
Day 1	94.68	92.97
Day 2	95.84	93.49
Day 3	94.12	93.71
Day 4	93.41	92.26
Day 5	91.96	91.97
Day 6	93.42	93.22
Day 7	91.68	90.25

**Table 4:** Load forecasting accuracy (from April to May).

Forecasting object	Forecasting method of deep learning (%)	Existing methods (%)
Shuanglong station #2	96.66	96.41
Fangxia station #1	93.98	93.38
Gangcheng station #2	92.67	93.14
Huihe station #2	96.89	96.88

**Table 5:** Load forecasting accuracy (from June to July).

Forecasting object	Forecasting method of deep learning (%)	Existing methods (%)
Shuanglong station #2	97.07	96.61
Fangxia station #1	93.98	93.02
Gangcheng station #2	93.59	94.01
Huihe station #2	94.59	94.07

**Table 6:** Load forecasting accuracy (from October to December).

Forecasting object	Forecasting method of deep learning (%)	Existing methods (%)
Shuanglong station #2	97.74	96.38
Fangxia station #1	96.22	91.63
Gangcheng station #2	97.25	96.12
Huihe station #2	98.32	96.19

## Data Availability

The data set can be accessed upon request.
